# Leveraging a Neuroevolutionary Approach for Classifying Violent Behavior in Video

**DOI:** 10.1155/2022/1279945

**Published:** 2022-07-15

**Authors:** Carlos Flores-Munguía, José C. Ortiz-Bayliss, Hugo Terashima-Marín

**Affiliations:** Tecnologico de Monterrey, Escuela de Ingeniería y Ciencias Ave, Eugenio Garza Sada 2501 Sur Col, Tecnológico C.P. 64849, Monterrey, Nuevo Leon, Mexico

## Abstract

Security has become a critical issue for complex and expensive systems and day-to-day situations. In this regard, the analysis of surveillance cameras is a critical issue usually restricted to the number of people devoted to such a task, their knowledge and judgment. Nonetheless, different approaches have arisen to automate this task in recent years. These approaches are mainly based on machine learning and benefit from developing neural networks capable of extracting underlying information from input videos. Despite how competent those networks have proved to be, developers must face the challenging task of defining both the architecture and hyperparameters that allow such networks to work adequately and optimize the use of computational resources. In short, this work proposes a model that generates, through a genetic algorithm, neural networks for behavior classification within videos. Two types of neural networks evolved as part of this work, shallow and deep, which are structured on dense and 3D convolutional layers. Each network requires a particular type of input data: the evolution of the pose of people in the video and video sequences, respectively. Shallow neural networks use a direct encoding approach to map each part of the chromosome into a phenotype. In contrast, deep neural networks use indirect encoding, blueprints representing entire networks, and modules to depict layers and their connections. Our approach obtained relevant results when tested on the Kranok-NV dataset and evaluated with standard metrics used for similar classification tasks.

## 1. Introduction

Nowadays, violence harms people physically and mentally. Besides, it severely harms the economies of many countries. Violence and crime represent a problem that we all have to deal with. Unfortunately, while governments are trying to counteract insecurity, citizens continue to suffer from criminal violence. As an example, in Mexico, estimations based on the number of investigations initiated in 2019 indicate that the most common types of crimes include nearly 150 thousand cases of theft from 4-wheeled cars, more than 82 thousand cases of residential burglary (with and without violence), almost 83 thousand cases of robbery to passers-by on public streets, around 18 thousand cases of theft in public transportation, and over 118 thousand cases of robbery to businesses [1]. The types of crimes described above, added to the lethal records, motivate families and businesses to install security cameras in homes, parking lots, and public places, to mention some. Although crimes can occur anywhere, in this work, we focus on violent acts in public places such as streets, pavements, shopping centers, or schools.

Crime leaves psychological marks on its victims, which are unable to cope with using common psychological resources [2]. The latter causes various types of emotional sequelae that negatively affect their lives. Among the most common disorders we can mention negative feelings, anxiety, constant concern due to trauma, depression, progressive loss of personal confidence, decreased self-esteem, alterations in the heart rhythm, and insomnia [3]. Conversely, physical integrity produces other effects such as injuries, trauma, cuts, fractures, and more. Regarding physical violence, it is possible to identify the aggressor's actions by looking at the interaction between the aggressor and the victim (their actions and movements), which are observable for just a few seconds. Observing such interactions is the basis of our proposal.

A reliable video surveillance system should be aware of what is happening at a particular moment and the actions that could result in potentially dangerous situations [4]. Covering all events in most current video surveillance camera systems requires security workers to watch what happens periodically. One of the main disadvantages of this approach is the cost of keeping people working for so long, which is likely to cause human errors because of tiredness and fatigue. Even if we can overcome these issues, each observer may rate an individual's suspicious action differently depending on their criteria and experience. These differences may cause the detection of actual suspicious actions to take longer to be labeled as such and to avoid undesirable situations [5]. Detecting violent attacks, robberies, and other criminal conducts requires a change in video surveillance systems that adapts to the current requirements [6]. For example, Martínez-Mascorro et al. [7] proposed a video surveillance system powered by AI that allows the early detection of robbery attempts through the analysis of behavior. In their work, they classify video segments as normal or suspicious, where the latter is interpreted as an indication that a robbery is about to occur. As we can observe, the constant development of artificial intelligence algorithms seems like an excellent option when detecting different behaviors in people captured by video surveillance cameras, which is the focus of this work.

Current research uses different techniques based on deep learning to tackle problems for image/video pattern recognition such as 3D convolutional neural networks [8–10], hybrid architectures using convolutional neural networks, and long-short term memory [11, 12], or including any form of deep learning for feature extraction, transformation, or classification at some point in their pipeline. However, their use may be limited because the topology of the neural networks is fixed. Therefore, the number of nodes and hidden layers must be chosen, leading to questions such as: how many hidden layers and hidden neurons per layer should the networks have? How many training pairs should the training phase use? Which neural network architecture is the best? Finding the values for the parameters is one of the most important steps because failing to do so usually causes the neural network not to be powerful enough to meet the requirements [13] or increases the error by accuracy saturation [14].

Neural network developers usually answer the above questions using their previous experience and design a fixed architecture throughout the training. On the opposite, in nature, the human brain has evolved up to 100 billion neurons and 100 trillion connections. This number surpasses, by far, the number of neurons and connections our ancestors counted with [15]. Similarly, hyperparameters in artificial neural networks should change in time by leveraging the ancestors' knowledge.

Neuroevolution is a type of artificial intelligence inspired by the evolution of biological nervous systems, used to generate artificial neural networks with a suitable topology and parameters to perform a given task. Neuroevolution has proved to be a reliable alternative in different tasks such as the classification of the electrocardiographic signal in health applications [16], the design of mobile robot controllers in robotics [17] or in video games to play at a human-like level [18]. However, detecting violent behavior in videos through neuroevolution remains an unexplored topic. Given the good results of neuroevolution in different scenarios, we consider it may also achieve competent results for generating networks that correctly classify the behavior shown in a video as violent or normal.

In this work, we are motivated by the idea that by providing tools that allow for the prompt detection of violent behavior, we can help people maintain a safe environment and respond accordingly to such stressful situations. Then, we address the problem of creating a suitable architecture for a neural network to classify behavior in videos correctly. For this purpose, we use genetic algorithms to create and evolve neural networks that, without human intervention, recognize violent-related activities in people who appear in the range of vision of a surveillance camera.

To summarize, the main contributions of this work are as follows:

1. Advancing towards surveillance systems that rely less on human intervention since our system can adequately discriminate violent behavior from a normal one in video clips from the database used for this work.
2. Contributing to the automation of designing neural networks since we use a genetic algorithm to generate different architectures of neural networks to detect violent-related activities in videos.
3. Providing empirical evidence that both dense layer–based and 3D convolutional layer–based networks can sidestep the task of detecting violent-related activities in videos.

The remainder of this document is organized as follows. In Section 2, we introduce different approaches from the literature that address the detection of different behaviors, as well as related works on the evolution of neural networks.  Section 3 describes the technical overview of different methods used in this work for evolving neural networks. The dataset, the procedure to extract features from videos, the fitness function, and the metrics considered in this work are detailed in Section 4.  Section 5 presents the experiments and results of the proposed approach for generating shallow, deep dense-based, and 3D convolutional neural networks, respectively. Finally, Section 6 presents the conclusion and some ideas for future work.

## 2. Related Work

This section describes relevant works that are significantly related to the problem we address and how we solve it in this work. We first describe the problem and emphasize how current solving approaches are limited since they depend on human intervention. Later, we describe different solving approaches described in the literature, which cover systems using spatiotemporal features, pose estimation, and deep features. We finally describe neuroevolution and NEAT as a way to familiarize ourselves with the rationale behind this work.

Intelligent video surveillance systems are based on observable behavior monitoring, categorizing it into different classes. For instance, we can mention theft, violence, and fraud detection, among others [19]. Existing intelligent video surveillance systems for behavior classification generally fall into one out of three broad groups, according to the set of features used to classify: two-dimensional, three-dimensional, and deep features. Among these categories, two-dimensional recognition systems have been explored the most [19].

Systems using two-dimensional features employ spatial information and RGB intensity to classify the cases. One example of such systems was proposed by Li et al. [20]. Their system relies on analyzing spatiotemporal video-volume space configuration to detect and localize anomalies in videos. Their method considers three main steps. The first step is the construction of an activity codebook through the extraction of low-level features referring to the global activity patterns on the video. The second step detects the anomalies at local sites using a Bag-Of-Words approach on a video cube (a spatiotemporal video window), producing composition-representation vectors. The third, and final step, builds a dictionary to detect the video activities and locates the regions where anomalies occur.

Another example using 2D spatiotemporal features involves two optical flow-based motion descriptors in Ref. [21]. The authors propose two spatiotemporal approaches to solve the detection of abnormal activities. The first one, called Silhouette and Optic Flow-based Features (SOF), uses background subtraction, then the optic flow values are generated. On the other hand, the second motion descriptor uses the Dense Trajectory Based Features (DTF), a method that calculates trajectories to create Histogram of Gradients (HOG), Histogram of Optic Flow (HOF), and Motion Boundary Histogram (MBH) descriptors, followed by a standard bag of visual words approach to create a visual vocabulary (codebook). Both SOF and HOF use a one-class Support Vector Machine (SVM) classifier to classify normal and abnormal samples. The two methods proposed endure major drawbacks despite promising results. As in most real-life scenarios, these methods can work well in a particular dataset, but their performance worsens in others. This is a problem that is present in real-life implementations. Not all the scenarios will be the same, yet the algorithm must generalize to be distributed in different environments and work acceptably.

Methods employing two-dimensional features typically use speed, direction, trajectory, and optical flow to understand the behavior of the entire scene captured by a camera. However, these characteristics apply to the people in the scenes and the elements that move in the videos. Thus, objects falling, rolling, or other elements that work by moving on their own can cause noise in the evaluation of scenes. Moreover, changes in lighting, reflection, or background clutter can significantly affect the method's performance. One way to better understand the movements relies on skeleton-based features. These approaches tend to have better results because they are less limited than previous ones. It is better to use the shape of the poses as well as their deformations over time to understand the silhouette of a person similar to real life, rather than just the representation of the two-dimensional segmentation approach that would consider a binary image silhouette [22].

Therefore, the pose estimation approach is gaining strength among researchers despite the need for better hardware. For example, Markovitz et al. [23] interpret people's poses using graphs to mitigate the viewpoint and lighting problems of the scenes. Weighted adjacency matrices generate pose graphs where each node represents a key point, a body joint, and each edge represents some relationship between two nodes. Some implementations work with skeletons at the cost of using additional devices. For example, Chaaraoui et al. [24] use Microsoft's Kinect since this type of RGB-D device has become cheap over the years and offers remarkable results in retrieving information from human bodies. They propose a novel skeletal-based spatiotemporal feature called the Join Motion History feature (JHM), representing the 3D location of skeletal joints and motion's age. As a classifier, they use the Bag-Of-Key-Poses method described by Chaaraoui et al. [25].

To conclude, deep learning models produce classes based on deep features. Such deep learning models include convolutional neural networks (CNNs) and recurrent ones, which tend to have more embracing use in addressing problems of this kind. One example of such methodologies is described by Vignesh et al. [26], where a CNN is used together with Long short-term memory neural networks (LSTM) to classify between normal and violent behavior frames. The convolutional network learns the spatial features of the images, and the LSTM neural network learns the long-term dependencies between frames. The main disadvantage of this work is the extraction of spatial and temporal features as different models carry it out. Li et al. [8] use a 3DCNN model without the addition of handcrafted features or RNN architectures to avoid the need for two different models. Handcrafted features can be eliminated because methods focused on deep learning can yield robust results and great accuracy.

The works described above are built on hand-designed architectures. In most cases, the hyperparameters are defined and set based on the expertise of their designers. Various works based on genetic algorithms have dealt with the constructions of neural networks by minimizing human intervention. One example is described by Xie and Yuille [27] as a genetic CNN. They propose a direct encoding represented as a fixed-length binary string that, in turn, is split into stages trying to simulate the parts into which state-of-the-art models are partitioned. The most critical limitation of genetic CNN concerns the genome representation since a fixed-length encoding affects networks that need to be deeper in order to converge to global (minima/maxima) values of the solution space. Besides this, the kernel size is also fixed within each stage. This limitation can help prevent networks from growing out of control and restrain the search space's size.

Large-Scale Evolution of Image Classifiers [28] overtakes the disadvantages of the previously detailed approach with fewer restrictions in depth, arbitrary connections, and numerical parameters by relying on individual encoding as graphs called DNA. The authors predefined a set of operations, similar to human designers' actions when constructing a network, which can be carried out on the mutation step as Remove-Convolution, Alter-Stride, Filter-Size Alter-Number-of-Channels, Add-Skip, and more. Authors of Large-Scale Evolution of Image Classifiers emphasize the massively parallel computational power required by their work. Nevertheless, some works seek to optimize resources. For example, Efficient Multi-Objective Neural Architecture Search via Lamarckian Evolution [29] proposes a multi-objective evolutionary algorithm for architecture search. This multi-objective function allows an approximation to the Pareto front (a front of solutions dominating all other solutions), optimizing several objectives such as accuracy, size of the network, and number parameters. To avoid large resource consumption, the authors choose individuals that most fit the Pareto front using the set of cheap objectives (easily calculable objectives such as the number of parameters) and evaluating this subset on their expensive objectives, in addition to employing a Lamarckian inheritance where learned parameters are passed to network's offsprings.

Initial approaches for neuroevolution are based on direct coding. The genome treats each node and connection as an individual element, making it more difficult and memory-consuming to store all of them in the population during the evaluation of generations. Another disadvantage of this idea is that it cannot reuse elements and must be coded and evolved independently. The Hybercube-based NeuroEvolution of Augmenting Topologies (HyperNEAT) [30] uses Indirect Encoding employing a variant of an artificial neural network called a connective Compositional Pattern-Producing Network (CPPN) [31], which represents sophisticated repeating patterns in the Cartesian space. These CPPNs produce spatial patterns based on functions such as Sigmoid, Gaussian, Sine, Cosine, Tanh, Relu, and others to exhibit properties of all these activations and create a symmetrical output, a repeating pattern, a repeating pattern with variation, and more. These patterns can be produced thanks to spatial interpretations of patterns generated within a hypercube (hence the name) as connectivity patterns in a lower-dimensional space. The CPPN does not work as a neural network for inferring based on the input data. Instead, it generates the weight of the connection between two neural network nodes being searched. It receives the coordinates of the Cartesian space between two nodes located in an *n* -dimensional space called the substrate.

However, HyperNEAT also presents some disadvantages. The most obvious one concerns the positions the hidden layer nodes should have. This is a decision that must be made by the developer as CPPN is not able to determine them, although there is an extension to HyperNEAT called ES-HyperNEAT (evolvable-substrate HyperNEAT) [32] which looks for areas with much variance in the pattern produced by CPPN, and it remains costly in execution time.

In this work, we propose using NeuroEvolution of Augmenting Topologies (NEAT) and its extension, Co-Evolution Deep NEAT (CoDeepNEAT), to solve the task of detecting people comparing two different types of networks: shallow and deep ones based on dense and 3D convolutional layers. These networks were selected as they do not carry over other approaches' problems and solve previously untackled problems (like the co-evolution of different niches).

## 3. A Brief Review on NEAT

The literature describes several works on the creation of neural networks through an evolutionary process [33, 34]. Such works can be divided into two large groups based on the encoding they use [35]. The methods that rely on direct encoding use the genome to establish the network topology within the phenotype. Usually, the representation relies on binary encoding to represent the neural network connections. However, this method is limited to the size of the matrix used to store the bits [34]. The second group is formed by the methods that use indirect encoding. These methods rely on rules to precisely indicate how the phenotype—that is, the neural network—will be constructed based on such rules. The most significant problem with this type of encoding is that it does not directly map the information from the genotype into the phenotype (the neural network), which may move the search away from desirable solutions. In this work, we evaluate two different types of neural networks, Shallow networks generated by NeuroEvolution of Augmented Topologies (NEAT) and Deep networks evolved by CoEvolution Deep NEAT (CoDeepNEAT). The overall technical explanations of these techniques are given as follows.

### 3.1. Neuroevolution of Augmented Topologies (NEAT)

Genetic algorithms have applications in many fields, including Neural Networks. NeuroEvolution of Augmented Topologies (NEAT) [36] has been used for reinforcement learning problems and has even proven to perform better than other reinforcement methods like Adaptive Heuristic Critic for solving the single-pole balancing problem [37].

Using a direct encoding for evolving neural networks is difficult because of the different components involved in an artificial neural topology, such as the number of neurons and connections. Instead, NEAT encodes each genotype with two lists, one for storing all the nodes (called *node genes*), which includes inputs, hidden and output nodes in the neural network, and a second one (*connection genes*) that represents all the connections between every pair of nodes as seen in Figure 1. Each of the nodes in the node genes has two attributes, one node number and the other for the type of node it represents (which can take a value from *Sensor* (Input), *Output,* and *Hidden*). On the other hand, the elements in the list of connection genes have more than two attributes specifying the in-node, out-node, the weight of the connection, a Boolean pointing if it is enabled or not, and an innovation number allowing finding its corresponding genes. A visual representation of these genotypes and phenotypes is shown in Figure 1.

The innovation number of each element in the list of connection genes allows NEAT to use information in the historical origin to perform crossover. When two networks are selected for crossover, they are lined up following the gene's historical markings producing *matching genes*, and *disjoint genes* referencing nodes and connections being removed or kept in a new neural network. Moreover, mutation and crossover could lead new individuals' fitness to drop and lead them to a lower probability of survival even when these mutations can significantly help future generations. This is the reason why NEAT uses *speciation* acting like a niche, where individuals are only allowed to compete with others in the same niche.

### 3.2. Coevolution Deep NEAT (CoDeepNEAT)

Just like HyperNEAT, CoDeepNEAT is also another extension of NEAT [38, 39]. NEAT is first extended to deep neural networks by calling it “DeepNEAT” using the same principles: individuals of minimum complexity are represented as graphs, nodes and edges are added or removed using mutation, and historical markings are used during crossover to align individuals and combining them among the most similar ones, the population is divided into species based on a similarity measure and each species grows proportionally to fitness with evolution occurring separately in each species. The main difference to NEAT is that it does not evolve complete networks; each individual is represented as a graph, and each node represents one or more layers of the deep neural network. In addition to these layers, each node also contains a table with hyperparameters, known as “node hyperparameters,” containing real or binary values mutated through evolution via a random bit-flipping (using a uniform Gaussian distribution) depending on the type of value. Those also help identify the type of network (convolutional, fully connected, recurrent) and properties such as the number of neurons, kernel size, and activation function. The edges no longer indicate weights but with which other layers they are connected to.

The graph also has a table called “global hyperparameters” that, as the name suggests, describes the hyperparameters that apply to the entire network, such as training algorithm, learning rate, and data preprocessing steps. DeepNEAT tends to produce complex and unprincipled structures, and CoDeepNEAT solves this by evolving two different populations of blueprints and modules separately.

Blueprints refer to graphs representing individuals where each node points to one subpopulation or species of modules. Each module is a graph representing a small DNN. When the evaluation of a generation starts, the blueprints replace the node with a module to the species it points to, as illustrated in Figure 2, and the hyperparameters in the “node hyperparameters” table are applied. Once the network is assembled (when all the nodes were replaced by their modules), the “global hyperparameters” table is also applied, and the evaluation starts. The overall fitness of the network is attributed back to blueprints and modules as average fitness. This evaluation reduces noise and allows blueprints or modules to be preserved for future generations even when they performed poorly in an assembled network. Once CoDeepNEAT ends, the best network is trained until it converges and is evaluated using a different test set.

## 4. Dataset, Features, and Metrics

Features used to feed the networks are an essential part that should be carefully chosen as they help the models to converge faster with the best inference results. The dataset and how the features were obtained from the videos are described in this section. Moreover, the fitness function (how well an individual performs during the training) and the evaluation metrics (how well each model performs on unseen data) are also described in their corresponding subsection.

For a reference, Figure 3 provides a general view of the pipeline proposed for evolving shallow and deep neural networks followed in this work.

### 4.1. Kranok-NV Dataset

This work uses the Kranok-NV dataset to evolve and train neural networks. The Kranok-NV dataset [40] consists of 2,026 videos, divided into 597 violent behavior videos and 1,429 normal behavior ones with a resolution of 840 pixels width and 472 pixels height, each having a different duration. This dataset was built for explicit use for violence detection in classification tasks. Violent behavior videos were made up from the YouTube website of people training in different practices such as boxing and kickboxing in joint or individual activities. In contrast, normal behavior videos consist of people going from one place to another walking down a corridor from three different cameras/angles in a closed-circuit television camera system. There is a noticeable class imbalance in the number of videos in the dataset. However, violent behavior videos have more frames as a whole than normal behavior videos because of their length. The class with fewer instances (normal behavior) was upsampled using two different techniques: zoom and mirror. The camera's vision field gets smaller by using zoom but makes objects (including people) bigger. Mirror comprises a horizontal flip in the image leaving, for instance, people that went from left to right now going from right to left. In addition, 5-fold Cross-Validation was used in the training phase partitioning the dataset into five equal-sized subsamples trying to keep as close as possible to 50/50% class balance in the number of frames. Kranok-NV is freely available at https://www.kaggle.com/kevinbkwanloo/kranoknv.

### 4.2. Feature Extraction

Previous works not based on neural networks have based their solutions in features like binary image silhouette [22] or in histograms of gradients [41], among others. This has been done regardless of whether such features represent people and may represent other noisy elements. Furthermore, those features do not directly represent attributes for behavior classification. Instead, they tend to represent the entire scene. Thanks to machine learning advances, human pose recognition has also had advances in different areas, even going from 2D output of human pose estimation in images to 3D shape–based on RGB-D devices and estimation from video. In contrast to the former described features, poses map actions of people that humans can easily interpret, so a network is expected to do the same.

There are many types of research related to pose estimation in which the detection and estimation of people's poses are made in a short time with high accuracy. In this project, such a task relies on deep learning models. Deep learning models for human keypoint detection are classified into two groups, depending on the order of the operations of the approach; top-down and bottom-up, bottom-up models are more robust to occlusion and complex poses. For instance, OpenPose [42–45] is defined as a *multi-person real-time keypoint detection* and operates as a bottom-up approach and was (and continues to be) one of the best alternatives for pose estimation. Nevertheless, it requires high-end GPU hardware to run correctly at competent Frames Per Second in live videos, like those in closed-circuit television environments. Fortunately, there are other options, such as Lightweight OpenPose [46], which is the one used in this work. The authors designed this option intending to maintain the excellent inference results but make it more suitable for real-time performance on edge devices, not only to be run in a GPU but also usual CPUs.

Two out of three neural networks evolved in this work share the same features. Shallow and deep neural networks based on dense layers expect numerical values as input in their input layers, leading to the same data for training and testing. In contrast, 3D convolutional neural networks expect images represented as numerical values in a 3D vector (height, width, and channels), requiring a particular feature preprocessing step. Nevertheless, a single pose cannot provide enough evidence about people's behavior considering a person could have a pose similar to another different action and be classified as such. We can use the poses' keypoints as spatial features plus their evolution throughout frames to extract the context as in Figure 4. This is achieved by stacking the poses from previous frames and iteratively keeping track of them. The angle between keypoints determines the spatial features. This is utilized to avoid using the raw Lightweight OpenPose's keypoints output and help offer a better generalization in the features. Such angles are calculated by using the arctan formula.

On the other side, temporal features are added by taking the person's pose in the video and seeing how the pose evolves in time. The longer the period, the more complex the neural network should be. Nevertheless, shortening the length of the period to reduce the network complexity may seriously decrease its classification power. The process for tracking people is described in more detail in Section C. Thus, measuring the relations in the people's poses and tracking their change over a short period (ten frames) can perfectly describe their behavior and be mapped to a classification using a neural network.

All the preceding describes the features used to input shallow and dense neural networks. Nonetheless, the feature extraction for 3D Convolutional Neural Networks (3DCNNs) is simpler. This is mainly attributable to 3DCNNs having the skill to model complex, both spatial and temporal, characteristics using cube-shaped kernels [9]. Experimentally, 3DCNN should outperform models with handcrafted features as long as the feed sequences are of correct data related to the task to be solved. Therefore, only video sequences with people in the field of view must be used in training and real-time implementations. Consequently, noise in the training data refers to every sequence not containing people, primarily if that sequence comprises objects in movement, although frames with no people can be labeled as nonaction.

3DCNN receives a 10-frame sequence as a context span to maintain a similarity in time concerning the input of shallow and deep dense networks. As previously stated, only if there is at least one person in the frame, then that frame can be used as part of the sequence. However, if there are no people in the frame, it cannot be used as part of the sequence nor past frames where people did appear. Thus, the entire sequence is discarded. Both features, pose angles based on pose estimation and video sequences, use ten frames as the pose's context, and networks do not receive noisy frames without people. In conclusion, the algorithm somehow trains all the networks with the same features.

Overall, a brief description of the previously detailed feature extraction step is detailed in the data preprocessing stage depicted in Figure 3.

### 4.3. Tracking

Tracking employs the keypoints of the people's poses to simulate the skeleton as independent variables to feed the networks. As mentioned before, in this work, we use Lightweight OpenPose [46] as a pose estimator. The neural networks should classify human actions based on their pose with such a skeleton. Conversely, a single pose as the context may attribute multiple false-positive classifications given that it could match with another pose of a different activity as someone moves. Thus, additional context is essential and should also be fed into the network and the pose. The temporal features are extracted by concatenating a sequence of poses as long as the person appears in the video sequence (tracking).

The approaches for detecting and tracking people are usually separated into two categories: Model-Free-Tracking (MFT) and Tracking-By-Detection (TBD). Tracking-By-Detection trackers are more widely used nowadays. Such models have several advantages, such as not requiring people in the first video frame, dealing with many people in the image, high detection accuracy, and not accumulating minor errors resulting in significant performance degradation in long videos. The solution comes by localizing the target in each frame without reliance on previous inferences. Instead of adding a new model on top of our solution approach, we decided to perform the tracking task using only the keypoints extracted by Lightweight OpenPose. The operation works by associating each person based on their whole body comprising joint points with a unique identifier on the first frame the person appears in the image. On posterior frames, each individual is compared with every person in the previous frame using their area of interest/bounding box by an operation called Intersection-over-Union (IoU), chooses the one with the highest rate, obtains its ID value, and assigns it back as its current ID will allow us to track their poses over time.  Figure 5 shows a visual example of applying IoU.

### 4.4. Fitness and Evaluation Metrics

Fitness must be assigned to each individual in the population over generations. Although we could have chosen the model's accuracy as a fitness value, it does not consider the class imbalance, and then, it does not penalize large errors in the classification. Fortunately, Shallow, Deep Dense, and 3DC neural networks use the same loss function, which does take large errors into account. Categorical Cross-Entropy was chosen as such a loss function given this task is a classification task using a one-hot encoded output.

We have opted for five popular metrics used in many classification applications. These metrics are defined below.

(1) $$\begin{array}{c} \text{Accuracy}=\frac{\mathrm{TP}+\mathrm{TN}}{\mathrm{TP}+\mathrm{FP}+\mathrm{FN}+\mathrm{TN}},\\ \text{Precision}=\frac{\mathrm{TP}}{\mathrm{TP}+\mathrm{FP}},\\ \text{Recall}=\frac{\mathrm{TP}}{\mathrm{TP}+\mathrm{FN}},\\ F1=2*\frac{\text{Precision}*\text{Recall}}{\text{Precision}+\text{Recall}},\\ \text{Specificity}=\frac{\mathrm{TN}}{\mathrm{FP}+\mathrm{TN}},\\ \text{Balanced accuracy}=\frac{\text{Recall}+\text{Specificity}}{2}. \end{array}$$

In all cases, TP, FP, TN, and FP stand for “true positives,” “false positives,” “true negatives,” and “false positives,” respectively. All these values can be extracted from the corresponding confusion matrices. It is relevant to recall that the values for Precision, Recall, and F1-score obtained from a confusion matrix when violent behavior is the class of interest may change when the class changes to normal behavior. Conversely, the accuracy and balanced accuracy do not change when the class of interest changes.

## 5. Experiments

In this section, we describe the experiments conducted and the results obtained.

### 5.1. Evolution of Shallow Neural Networks through NEAT

This section describes the NEAT implementation and how we incorporated it into the training of the shallow neural networks. We have selected a set of hyperparameters that produce an acceptable performance of the genetic algorithm on each fold. These hyperparameters were obtained by preliminary experimentation, running the algorithm several times until finding the ones that perform satisfactorily on different scenarios.

It is well known that, for genetic algorithms to work correctly, they require to tune many hyperparameters, such as initial population size, initialization of individuals, probabilities for mutation, crossover, and more. A slight modification of these may lead to drastic changes, for better or for worse. Several runs of the NEAT-based part of this work were conducted to find the best configuration of hyperparameters for producing the neural networks. The selected configuration considers running for 100 generations, where the probability of adding or deleting a connection between nodes is 50%, respectively. Besides, the probability of adding and deleting a node was 50% for each case. Lastly, only the two best individuals from each species remain untouched and are moved to the next generation, while 20% of each species is allowed to reproduce.

When an individual is initialized, a connection between input and output nodes is established, with a 50% probability. This means that, on average, each individual starts with half of its input nodes connected to half of its output ones. The former was done to avoid starting with completely disconnected neural networks (individuals), which may increase the algorithm's convergence time. Finally, the neural network has two output nodes representing violent/normal behavior, with a softmax postprocessing. The results presented in this section correspond to one network out of the 100 produced (the one with the highest fitness) using ten frames as input.

Figure 6(a) presents the confusion matrix of the Shallow neural network when violent behavior is the class of interest. 245,874 (48.95%) samples were correctly classified as violent behavior, while 221,750 (44.15%) samples were correctly classified as normal behavior. The larger the TP and TN in a confusion matrix, the better the network's performance (they represent the successes). Thus, the Shallow neural network performed notably, obtaining an overall accuracy of 93.6741%.

As we mentioned before, the values for Precision, Recall, and F1-score depend on the class of interest. Although both types of behavior are relevant, it is critical to identify violent behavior over the normal one in this work.  Table 1 shows the results of Precision, Recall, and F1-score for both violent and normal behavior. Although the performance is similar in all the metrics, for Precision and F1-score, the Shallow neural network was slightly better at identifying violent behavior than the normal one.

As observed from Table 1, the Shallow neural network seems to exhibit a well-balanced behavior. A balanced accuracy of 93.7111% confirms this. Overall, the Shallow neural network performed well for classifying the video samples as violent or normal.

### 5.2. Evolution of Deep Neural Networks through CoDeepNEAT: Dense Layers

The following model is an extension to evolve deep neural networks to detect violence in videos. There is a similarity between the shallow neural network evolved using NEAT, and the dense, deep neural networks evolved using CoDeepNEAT: how input values are fed into the networks. Both models expect feature vectors representing ten frames of angles between joints from the body of people in videos; therefore, both models use the same dataset for training and testing along with 5-fold cross-validation.

The hyperparameters for the macro and micro-architecture, i.e., the Blueprints and Modules, respectively, were selected after several runs and are described as follows. The blueprints' hyperparameters are set and not modified throughout the evolutionary process. Such hyperparameters include the loss function using *categorical cross-entropy*, Adam optimizer, along with its learning rate with a fixed value of 0.005. The output layer activation function is softmax right as in the shallow model approach described in the previous experiment. The only parameter we can vary is the number of nodes in the blueprint; it was set to three as a maximum and one as a minimum.

The modules' parameters (dense layers that will replace the blueprint nodes) comprise some nodes in a layer, in a range between 35 and 80, and activation and function, either ReLU or Sigmoid. In addition, each module can have a maximum of three dense layers and a minimum of one. In this manner, considering that the blueprint could have three modules as maximum and each module three layers, the largest neural networks produced by the algorithm would contain nine hidden layers. Nonetheless, the depth is extended by placing fixed layers at the beginning (after the input layer) and the end (before the output layer) of each blueprint. These fixed layers are used by reasoning that layers should have fewer nodes the closer to the output layer. Such fixed layers do not belong to any niche module. Instead, they are placed in their respective places at the beginning of the evolution process when the blueprint population is created and not removed or modified. One of these two “fixed” layers is contained after the input layer and can have node units ranging from 150 to 200 using a Sigmoid or ReLU activation function. The second “fixed” layer follows the previous one and can have node units from 80 to 120. All the modules (evolved in niches through the generations of the genetic algorithm) come after this second fixed layer, allowing the network to grow initially and eventually become more condensed towards the output. Furthermore, each dense layer in the modules is followed by a dropout layer using a rate from 0 to 0.07 units to drop. This helps the network to prevent from growing so much and producing overfitting.

The genetic algorithm runs for 20 generations using a population size of 15 blueprints and 30 modules, both evolving within their related niches. When possible, niches group similar blueprints and modules in three different species using the *k*-means clustering algorithm. Evolutionary parameters cover mutation set to 50% probability, crossover rate of 20%, elite modules and blueprints of 20%, the latter referring to keeping a portion of chromosomes intact and passing the individuals to the next generation without modifications.

Fitness is assigned when the blueprint's nodes are replaced with the respective modules niches they point to. One thing to look out for is that training each network using the entire dataset in every generation is computationally expensive and time-consuming. Therefore, only a portion of the dataset's training and testing data are used. For the fitness assignation, the networks are first trained using five training epochs with randomly picked samples equivalent to only 40% of the training data, and the fitness is yielded by the loss using 30% of randomly picked samples from the test set. Finally, the algorithm outputs the networks with the highest fitness and is converged using the entire training set during 15 epochs; its parameters are saved, and the classification results are presented in the section below.

As can be seen in Table 2, the metrics of the evolved networks using 5-fold cross-validation for ten frames as inputs outperform those from the Shallow neural network developed in the previous experiment. The deep dense neural network performs slightly above 98% in the same metrics used to evaluate the shallow network. From the confusion matrix depicted in Figure 6(b), we can observe that the overall accuracy has increased to 98.7333%. Moreover, the value of 98.7228% in the balanced accuracy confirms that this neural network maintains its quality across the two classes of interest.

### 5.3. Evolution of 3D-Convolutional Neural Networks through 3D-CoDeepNEAT: 3DCNN

So far, two types of neural networks have evolved: shallow and deep based on dense layers (also known as fully connected layers) using NEAT and CoDeepNEAT. The input values of these two types of networks are temporal features that indicate how the angles between joints change in a span of ten frames. However, the spatial features must also be considered to classify the activities. Convolutional neural networks (CNN), also known as Shift Invariant or Space Invariant Neural Networks, are highly used for this task, considering they are skilled at recognizing patterns in the input images by producing abstractions that are visible in activation maps. In short, the input images are feed representing low-level features, and the CNN is responsible for obtaining high-level features as data travel across the network.

CoDeepNEAT was developed to evolve convolutional neural networks. In this work, we have extended its functionality. We have seen that CNNs are better than fully connected and shallow neural networks for extracting the features from an image, although an iteration of CNNs adds one more dimension called 3D convolutional neural networks. As the name suggests, 3DCNN convolve cube-shaped kernels in a set of given images transforming their input into four dimensions; height, weight, number of channels, and sequence length. The sequence is conformed of *n* images stacked one after the other. The addition of images in the input eliminates the limitations of previous 2D CNN that convolve two-dimensional kernels into single images.

For the previous reasons, CoDeepNEAT was expanded to evolve 3DCNN and see if it can generate suitable architectures for these more complex networks. With that, the model addresses the same questions that arose with the previous models: how do we know that we have selected the architecture that gets the most out of our training data while at the same time generalizing to perform on previously unseen data?

Again, by using 5-fold cross-validation, the genetic algorithms will produce different models trained in different datasets, which will have unbiased error estimates on the test data. Many tests were conducted using a single fold from the five generated to select the most suitable evolutionary algorithm ratios such as crossover, mutation, number of elite individuals, generations, and the values of the hyperparameter tables of the nodes.

The definition of the final set of hyperparameters starts with the hyperparameters table, i.e., the blueprints. The table got the best results when the number of nodes in each blueprint was a minimum of 1 and a maximum of 2; this is the only value in such a table that can vary during the algorithm's run. Moreover, categorical cross-entropy was used as a fixed loss function, given that we are still working with the same multiclass classification problem. Adam optimizer is another fixed parameter with its learning rate established at 0.005. The softmax activation functions in the last layer of the neural network converting the values to a probability distribution. Lastly, the size of the input consists of 10 frames.

On the side of the modules, several values change in a uniformly random fashion. For example, the first *fixed* convolution layer (not included in modules) has as variable hyperparameters the number of filters/kernels that can range from 24 to 32 and the activation function deciding between either ReLU or Sigmoid. It is worth pointing out that it is the only layer that can have a max-pooling 3D compliment because arbitrary connections between layers are allowed, which means that some can be connected to more than one hidden layer. The problem emerges when some hidden layers get input values from more than one layer, which would cause incompatibility in the size of the inputs if the data come from a layer performing max-pooling while others do not. The output is concatenated to be compatible when two hidden layers point to a single layer.

Moving onto the hidden layers, they consist of numerous filters that range from 32 to 64. These filters use kernels of sizes 1, 3, or 5, with activation functions ReLU or Sigmoid. The layers' complement is dropout with a ratio from 0 to 0.5, avoiding overfitting, similar to the dense layer model evolved before.

The blueprint also contains two dense layers at the end of the architecture to help in the classification. A final dense layer is added after the nodes of the blueprint, containing between 490 and 600 nodes, with ReLU being the only activation function it can select from. The second dense layer is the last and is in charge of classifying if the behavior is normal or violent. The maximum number of layers for the modules is 2, while the minimum is 1. Thus, the maximum number of nodes in the blueprint plus the maximum number of layers in the modules entail networks with a max depth of four layers, without counting the fixed layers at the end and add-ons of each layer.

The evolution parameters are ten generations and a population of seven individuals. The number of blueprints and modules is seven too. Blueprints and modules are separated into three different species, each using *k*-means unsupervised classification algorithm. The crossover and mutation rates were set to 20% and 50%, respectively. Also, 20% of the population was allocated as the elite to keep the blueprints and modules without changes from one generation to another. The networks are trained using only 40% of the training data for four epochs, while 30% of the test data assign the fitness. The testing and results section presents the findings on the evolutions using 5-fold cross-validation with 10-frame inputs.

It is essential to highlight that the 3DCNN is a classifier of the whole video image which means it does not designate a probability rate to each person in the image. The entire frame (taking as context the previous nine) is classified as violent when the disturbance starts, opposite to the shallow and dense layer-based network models where each person was classified based on their own behavior and pointed using bounding boxes. The results in Table 3 confirm the superiority of the 3DCNN, supported by an overall performance of 99% on all the metrics.

Finally, we can conclude that the 3DCNN produced obtained almost perfect balanced accuracy (99.9850%), which confirms that it is a suitable model for classifying violent and normal behavior in the videos considered for this work.

### 5.4. Discussion

The work presented in this document shows how the coevolution of blueprints and modules also works for evolving neural networks it was not intended for (convolutional neural networks and long-short term memory networks). This idea leads to a belief that coevolution may also produce hybrid architectures. In addition, allowing arbitrary connections between layers shows that features extracted in previous layers can also help in attribute transformation on further layers. The previous practice is probably the most challenging part if a developer wants to build an architecture with skip connections at hand because one is unsure which intermediate layer would connect to the other.

However, as seen in the accuracy of the best individuals and population in CoDeepNEAT, the best individuals start with high accuracy since the beginning of the generations, which raises the question: is the genetic algorithm helping to find the best architecture? Cannot we just choose the best individual from the first generation avoiding the time of evolving the population? The short answer, according to our experiments, is no. The evaluations are performed using a different small portion of the dataset of each generation, so the initial architectures may fit that data well but may not do so well on the entire test set. The minor improvements of the best network (and the population in general) through the generations help generalize appropriately on the test set. Moreover, at the end of each run, almost all the individuals in the population reach the global optima, which confirm that the genetic algorithm is working properly. This leaves us with the possibility of choosing the final network according to different criteria; the network with fewer parameters, the deepest network, or simply the one with the best accuracy.

The results also show that even a shallow network performs well in this task. These three models leave us with various options to choose from, according to different needs. When the computational resources are scarce, we can sacrifice some accuracy and go for a shallow neural network. As the resources become available, we can move to dense layer neural networks or 3D convolution-based neural ones.

## 6. Conclusion and Future Work

This work proposes using neuroevolution as an alternative to generate topologies and choose the best set of hyperparameters for a neural network to classify behavior as either normal or violent in a surveillance system. The comparison of results leverages the model's ability to evolve networks based on their depth and the type of input they receive.

Genetic algorithms can select the correct architecture of a neural network to detect violent behavior. These algorithms can produce shallow and deep neural networks based on dense and 3D convolution layers. All the models analyzed in this work can perform this task with high accuracy. However, a deeper network can extract more information from the input data, leading them to produce the best results. Although the genetic part of the process finds the best architecture, one limitation is that we still need to deal with the parameters of the genetic algorithm itself, with some of them being difficult to choose. The list of hyperparameters in neuroevolution includes the crossover, mutation, elite individuals rate, desired number of niches, number of nodes per layer, number of kernels per layer, activation functions to choose from, and more. Of course, the length of the hyperparameter catalog increases for deep learning neural networks compared to genetic algorithms. Still, it is ideal to continue looking for the best set because GAs search several parts of the solution space simultaneously, so a bit of change in the probabilities of any other hyperparameter may affect the entire population, implying stagnation in local optima.

Regardless of our efforts, there are some areas related to the neuroevolution of neural networks for behavior classification in videos that we have not explored and represent some paths for future work. For example, we can mention handling different objective classes. Instead of just classifying two types of behavior (violent and normal), future developments could focus on suspicion, protest, fainting, or harassment, to mention some. In addition, more work is needed regarding the dataset. Nowadays, the Kranok-NV dataset is limited to violent and normal behavior only. In order to explore the classification of other behaviors, we require to extend the dataset to incorporate the corresponding samples. Besides, future work may involve running the same experiments using a different, larger video dataset. In these future experiments, some hyperparameters may change on both the genetic algorithm and the neural networks.

Future work can also integrate a multi-objective search if accuracy is not the only target function. The multi-objective search would allow an approximation to the Pareto front (a front of solutions dominating all other solutions), which can optimize several objectives jointly. As a result, the list of objectives can be quite diverse, ranging from searching for the network with the lowest loss, the highest accuracy, the network with the lowest number of parameters, and estimators of the network's depth.

Finally, we are aware that we need to compare our approach against others from the literature. In this work, we compared three neural network models, all generated through their particular implementation of a neuroevolutionary approach. Our models were generated on Kranok-NV, which undoubtedly influences the outstanding performance of the models. So far, the literature includes only another model trained on this dataset. Kwan Chong Loo [40] proposed the Kranok-NV dataset, and our networks improve on such a model and obtain better results in various metrics. For example, Kwan reports values for Precision, Recall, and F1-score of 99.05%, 97.70%, and 98.37%, respectively, for the normal behavior class. When comparing the results against those obtained by our 3DCNN proposal (Table 3), we obtain better results on the three metrics. For the violent behavior class, a similar situation occurs. Reported results indicate values of 97.44%, 98.94%, and 98.19%. When compared again, the three metrics are outperformed by our 3DCNN proposal (Table 3). Unfortunately, a comparison against other models not trained in this dataset seems unfair since there is a risk of biasing the results to favor our proposal. We plan to compare the performance of our proposal against others from the literature as part of future work.

## Figures and Tables

**Figure 1:** Individual representation NEAT: genotype and phenotype.

**Figure 2:** Coevolution of blueprints and modules.

**Figure 3:** Pipeline for evolving shallow and deep neural networks.

**Figure 4:** Poses' context from time.

**Figure 5:** Example of IoU applied in videos.

**Figure 6:** Confusion matrices for the three networks evaluated. (a) Shallow neural network. (b) Deep dense neural network. (c) 3D Convolutional neural network.

**Table 1:** Precision, recall, and F1-score obtained by the Shallow neural network for both classes of interest (violent and normal behavior).

	Precision	Recall	F1-score
Violent behavior	94.8773	93.1110	93.9859
Normal behavior	92.3655	94.3113	93.3283

**Table 2:** Precision, recall, and F1-score obtained by the dense neural network for both classes of interest (violent and normal behavior).

	Precision	Recall	F1-score
Violent behavior	98.7226	98.8937	98.8081
Normal behavior	98.7456	98.5520	98.6487

**Table 3:** Precision, recall, and F1-score obtained by the 3D convolutional neural network for both classes of interest (violent and normal behavior).

	Precision	Recall	F1-score
Violent behavior	99.9773	99.9886	99.9830
Normal behavior	99.9907	99.9814	99.9860

## Data Availability

The Kranok-NV dataset is publicly available at https://www.kaggle.com/kevinbkwanloo/kranoknv.
